The article "Serum Expression of ESM-1, HMWA, and AGEs and Its Relationship with Disease Severity in Patients with Gestational Hypertension" was retracted in 2023. Reasons: signs of a paper mill; compromised peer review; unreliable results or conclusions.

# Serum Expression of ESM-1, HMWA, and AGEs and Its Relationship with Disease Severity in Patients with Gestational Hypertension

**DOI:** 10.1155/2021/9545857

**Published:** 2021-12-09

**Authors:** Yun Yan, Linlin Luan, Jieru Xu

**Affiliations:** Department of Obstetrics, Qingdao Chengyang People's Hospital, China

## Abstract

**Objective:**

The research is to investigate the expression and the relationship between serum endothelial cell-specific molecular molecule-1 (ESM-1), high molecular weight adiponectin (HMWA), and late glycosylation terminal product (AGEs) in patients with gestational hypertension.

**Methods:**

75 patients with pregnant hypertension who were treated in our hospital from June 2019 to June 2020 were selected as the case group, and 70 healthy pregnant women with pregnancy examination at the same period in our hospital were selected as the control group to analyze the changes in serum ESM-1, HMWA, and AGEs levels and the correlation with the degree of illness and their predictive value.

**Results:**

Serum ESM-1 and AGEs were significantly higher in the case group than in the control group. Serum HMWA was significantly lower than that in the control group (*P* < 0.05). The gestational hypertensive serum ESM-1 and AGEs was significantly lower than in patients with mild preeclampsia and severe preeclampsia. Serum HMWA was significantly higher than in patients with mild preeclampsia and severe preeclampsia. Serum ESM-1 and AGEs of mild preeclampsia were significantly lower than in patients with severe preeclampsia. Serum HMWA was significantly higher than in patients with severe preeclampsia (*P* < 0.05). The result of correlation analysis shows a positive correlation between serum ESM-1 and AGEs (*P* < 0.05). A negative correlation was observed between HMWA and the degree of illness (*P* < 0.05).

**Conclusion:**

Serum ESM-1, HMWA, and AGEs are abnormally expressed in gestational hypertension, are closely related to the degree of condition, and have important clinical significance for condition control.

## 1. Introduction

Pregnancy-induced hypertension is a common disease in pregnancy, which mainly occurs after 20 weeks of pregnancy. According to the survey, the incidence of pregnancy hypertension in China is 9.4%. Patients mainly face edema, proteinuria, and hypertension symptoms, which can lead to premature birth, postpartum bleeding, and other adverse pregnancy outcome. Furthermore, it can threat mother and infant life seriously [1]. Therefore, early prediction of disease and judging its severity contribute to early treatment and is of great significance for improving adverse pregnancy outcomes. ESM-1 is a novel marker associated with endothelial dysfunction, which is at normal levels in normal endothelial tissues. It is widely expressed in multiple cardiovascular diseases when levels of endothelial cells are elevated during periods of damage [2]. Adiponectin is secreted by adipocytes. When hypertension increases in pregnancy, its level decreased and leptin level gradually increased. HMWA is the endogenous hormone polypeptide secreted by adipocytes and plays an important regulatory role in fatty acid oxidation and endothelial function [3]. AGEs is heavily expressed in placental trophoblast and vascular endothelial cells, which can cause intracellular oxidative stress promoting substantial expression of inflammatory factors in hypertension during pregnancy [4]. However, the studies on the serum ESM-1 and HMWA associated with the occurrence of gestational hypertension are not enough. Therefore, this study is aimed at exploring the expression of serum ESM-1, HMWA, and AGEs in gestational hypertension as well as its relationship with disease severity.

The article "Serum Expression of ESM-1, HMWA, and AGEs and Its Relationship with Disease Severity in Patients with Gestational Hypertension" was retracted in 2023. Reasons: signs of a paper mill; compromised peer review; unreliable results or conclusions.

## 2. Research Methods

In this research, we selected 75 patients with gestational hypertension treated in our hospital from June 2019 to June 2020 as the case group. The age of the group is 20~37 years (average: 28.51 ± 2.50), the gestational weeks of the group were 6 to 22 weeks (average: 14.26 ± 2.62), the parity frequency is 1~4 times (average: 1.63 ± 0.31), and the body mass index was 23.47~26.89 kg/m^2^ (average: 24.58 ± 1.05 kg/m^2^). Among the patients, 22 had gestational hypertension, 35 had mild preeclampsia, and 18 had severe preeclampsia. Furthermore, 70 healthy pregnant women examined in our hospital were selected as the control group. The age of the group is 21~38 years (average: 28.46 ± 2.37), the gestational weeks of the group were 5~25 weeks (average: 14.31 ± 2.60), the parity frequency is 1~3 times (average: 1.61 ± 0.25), and the body mass index was 23.39~26.96 kg/m^2^ (average: 24.61 ± 1.09 kg/m^2^). General data showed no significant difference between the two groups and can be compared.

The inclusion criteria include the following: (1) compliance with the relevant diagnostic criteria of guidelines for the diagnosis and treatment of hypertension during pregnancy [5]; (2) patients without relevant treatment before admission; and (3) informed consent. The exclusion criteria include the following: (1) patients with abnormal cardiac function; (2) patients with abnormal glucose tolerance and chronic hypertension or being treated with steroids before pregnancy; (3) patients with severe infection disease; (4) patients with malignant tumor; (6) patients with abnormal blood system; (7) history of drug and alcohol abuse; and (8) multiple pregnancy.

The article "Serum Expression of ESM-1, HMWA, and AGEs and Its Relationship with Disease Severity in Patients with Gestational Hypertension" was retracted in 2023. Reasons: signs of a paper mill; compromised peer review; unreliable results or conclusions.

Fasting venous blood was collected in the morning of the second day after the two groups were enrolled. Centrifugation was carried out at a speed of 3000 R·min^−1^ with a centrifugation radius of 10 cm and a centrifugation time of 10 min. It is stored in the freezer at −20°C for detection after the upper serum was extracted. The levels of serum ESM-1, HMWA, and ages were measured by enzyme-linked immunosorbent assay. The kit is produced by Shenzhen Jingmei Biotechnology Co., Ltd. The instrument used was Toshiba GA800 biochemical analyzer, and operation was performed strictly according to the instructions of the kit.

SPSS 18.0 package was used to analyze the data. The data were represented by mean ± standard deviation (±s). We use a *t*-test, ANOVA for multiple group analysis, and Spearman's correlation coefficient to analyze the data. We use the subject working feature curve (ROC) to predict the value of serum ESM-1, HMWA, and AGEs. *P* < 0.05 stands for statistical significance.

## 3. Results

### 3.1. Comparison of Serum ESM-1, HMWA, and AGEs Levels between the Two Groups

The serum ESM-1 and ages in the case group were significantly higher than those in the control group. The serum HMWA was significantly lower than that in the control group (*P* < 0.05) as can be seen in Table 1.

### 3.2. Comparison of Serum ESM-1, HMWA, and AGEs Levels for Different Disease Severities

Serum ESM-1 and ages in patients with pregnancy-induced hypertension were significantly lower than those in patients with mild preeclampsia and severe preeclampsia. The serum HMWA was significantly higher than that in patients with mild preeclampsia and severe preeclampsia. As can be seen in Table 2, the serum ESM-1 and ages in mild preeclampsia were significantly lower than those in severe preeclampsia, and serum HMWA was significantly higher than those in severe preeclampsia (*P* < 0.05).

### 3.3. Correlation Analysis of Serum ESM-1, HMWA, and AGEs and the Degree of Hypertension in Pregnancy

We took the degree of illness as the dependent variable and serum ESM-1, HMWA, and ages as the independent variables. The results of correlation analysis showed that serum ESM-1 and ages were positively correlated with the severity of the disease (*P* < 0.05). There was a negative correlation between HMWA and disease severity (*P* < 0.05). The data is shown in Table 3.

### 3.4. Value Analysis of Serum ESM-1, HMWA, and AGEs in Predicting Gestational Hypertension

The ROC results show that the AUC of serum ESM-1 in predicting gestational hypertension was 0.701, the sensitivity was 81.52%, the specificity was 86.59%, and the cutoff value was 1.14 *μ*g/l. The AUC predicted by HMWA was 0.652, the sensitivity was 84.15%, the specificity was 87.58%, and the cutoff value was 4.33 ng/ml. Serum AGEs predicted an AUC for hypertension during pregnancy of 0.982, sensitivity is 85.35%, the specificity was 88.28%, and the cutoff value was 44.87 ng/ml. The AUC of joint detection is 0.992, the sensitivity was 89.67%, and the specificity was 91.24% (higher than detection alone (*P* < 0.05)). The data is shown in Figure 1 and Table 4.

The article "Serum Expression of ESM-1, HMWA, and AGEs and Its Relationship with Disease Severity in Patients with Gestational Hypertension" was retracted in 2023. Reasons: signs of a paper mill; compromised peer review; unreliable results or conclusions.

## 4. Discussion

Gestational hypertension is a common special disease in late pregnancy. It is one of the important causes of premature delivery, low birth weight, and perinatal death [6]. The pathogenesis of gestational hypertension is complex, which is mainly due to placental ischemia and vascular endothelial injury, increasing vascular permeability. Thus, it causes the leakage of body fluid and protein in pregnant women, reduces the charge barrier of glomerular filtration membrane, and leads to the increase of protein content in urine. Some patients can also cause other complications such as renal failure, which seriously threatens the lives of mothers and infants [7]. Therefore, looking for disease-related indicators and judging the severity of the disease are of great significance for disease control and improving the therapeutic effect.

Studies have shown that vascular endothelium can produce more bioactive substances and play an important role in regulating vascular function. Therefore, vascular endothelial injury will lead to pathological changes of gestational hypertension [8]. ESM-1 is a new marker of endothelial dysfunction and one of the factors to maintain the functional stability of endothelial cells. ESM-1 has a wide range of biological activities and participates in the process of cell adhesion, migration, and proliferation [9]. ESM-1 plays an important role in cardiovascular diseases. For example, it is highly expressed in patients with essential hypertension and unstable angina pectoris complicated with hypertension. It can be used as a marker for the early diagnosis of diseases [10]. In this research, the results showed that serum ESM-1 in patients with pregnancy-induced hypertension was higher than that in healthy pregnant women. The level of ESM-1 increased gradually in gestational hypertension, mild preeclampsia, and severe preeclampsia, and there was a positive correlation with the severity of the disease. Serum ESM-1 is highly expressed in pregnancy-induced hypertension, which may be involved in the pathogenesis of pregnancy-induced hypertension. Qiaohong and Cong [11] also showed that ESM-1 is highly expressed in fetal endothelial cells and maternal endothelial cells of placenta of hypertensive pregnant women, which can increase with the severity of the disease and reflect the severity of the disease to a certain extent. The physiological functions of adiponectin include anti-inflammation and antiatherosclerosis. Adiponectin is a cardiovascular protective fat factor and plays an important role in endothelial inflammatory response and lipid metabolism. Adiponectin can promote the metabolism of blood lipid and blood glucose, inhibit the degree of inflammation of blood vessel wall, enhance vasodilation function, and regulate the stability of blood pressure [12]. Studies have shown that HMWA as a cardiovascular protective factor can reduce blood pressure and reduce the risk of insulin resistance and type 2 diabetes. Therefore, it is speculated that the decrease of serum HMWA is related to the occurrence of gestational hypertension and can predict the outcome of the disease [13]. In this paper, the results showed that serum HMWA in patients with pregnancy-induced hypertension was lower than that in healthy pregnant women. The level of ESM-1 in patients with gestational hypertension, mild preeclampsia, and severe preeclampsia decreased gradually, and there was a negative correlation with the severity of the disease. We also found that HMWA is lowly expressed in pregnancy-induced hypertension, which can decrease with the severity of the disease and can be used as a marker to predict the level of the disease. The reason may be related to the influence of insulin resistance and inflammatory response [14, 15]. Previous studies have shown that ages can participate in the pathogenesis of gestational hypertension through oxidative stress injury and lipid metabolism disorder [16]. In this paper, the results showed that serum age in patients with pregnancy-induced hypertension was higher than that in healthy pregnant women and could increase with the severity of the disease, which was positively correlated with the severity of the disease. The studies have shown that the expression of serum ages is high in pregnancy-induced hypertension, which can be used as a marker to judge the severity of the disease. The reason may be that the occurrence of gestational hypertension can lead to the pathophysiological changes of vascular endothelium and ages can promote oxidative stress and intravascular inflammatory injury, change the morphology of vascular endothelial cells, thicken the vascular wall, and narrow the lumen, causing tissue damage, and eventually lead to pregnancy-induced hypertension.

The article "Serum Expression of ESM-1, HMWA, and AGEs and Its Relationship with Disease Severity in Patients with Gestational Hypertension" was retracted in 2023. Reasons: signs of a paper mill; compromised peer review; unreliable results or conclusions.

AGEs is formed by the nonglycosylation reaction of lipids and proteins and reducing monosaccharides. It can cause intracellular oxidative stress and regulate the expression of a variety of cytokines and growth factors. AGEs can also regulate the expression of a variety of cytokines and growth factors, reduce the production of matrix metalloproteinases, and be produced in large quantities in the case of high blood glucose level and osteoarthritis [14, 15]. Studies have shown that AGEs can participate in the onset of hypertension during pregnancy through oxidative stress damage and lipid metabolism disorders [16]. The results of this study show that serum AGEs is higher in pregnant hypertension patients than in healthy pregnant women and can increase with the severity of the disease and the degree of illness, suggesting that serum AGEs expression is higher in gestational hypertension and can be used as a marker to determine disease severity. The reason may be because the occurrence of pregnancy hypertension can lead to pathophysiological changes in the vascular endothelium and AGEs can promote oxidative stress and intravascular inflammatory damage, change the morphology of vascular endothelial cells, make blood vessel wall thickening, lumen stenosis, lead to tissue damage, and eventually lead to the occurrence of pregnancy hypertension. The ROC analysis of this study showed that the AUC of serum ESM-1 in predicting gestational hypertension was 0.701 and the cut-off value was 1.14 *μ*g/l. The AUC predicted by HMWA was 0.652, and the cut-off value was 4.33 ng/ml. The AUC of serum ages in predicting gestational hypertension was 0.982, and the cut-off value was 44.87 ng/ml. The AUC of serum ESM-1, HMWA, and AGEs was 0.992, which was higher than that of single detection. It shows that the combined detection has a higher value in predicting pregnancy-induced hypertension.

In conclusion, the abnormal expression of serum ESM-1, HMWA, and ages in patients with pregnancy-induced hypertension is closely related to the degree of disease, which is of great clinical significance for disease control. However, the sample size of this study is small, and the changes of various indexes before and after treatment are not observed. In the future, the sample size should be increased for in-depth research.

## Figures and Tables

**Figure 1:** ROC curves of serum ESM-1, HMWA, and AGEs predicting hypertension during pregnancy.

**Table 1:** Comparison of serum ESM-1, HMWA, and AGEs levels between the two groups.

Group	Example number	ESM-1 (*μ*g/l)	HMWA (ng/ml)	AGEs (ng/ml)
Case group	75	1.37 ± 0.52	3.51 ± 1.21	48.91 ± 3.41
Control group	70	1.01 ± 0.07	4.43 ± 1.29	39.78 ± 2.52
*t* value		5.743	4.431	18.230
*P* value		0.001	0.001	0.001

**Table 2:** Comparison of serum ESM-1, HMWA, and AGEs levels for different disease severity.

Group	Example number	ESM-1 (*μ*g/l)	HMWA (ng/ml)	AGEs (ng/ml)
Pregnancy hypertension	22	1.22 ± 0.47	3.85 ± 0.83	45.62 ± 3.44
Mild preeclampsia	35	1.35 ± 0.41	3.47 ± 0.82	48.79 ± 3.52
Preeclampsia	18	1.59 ± 0.45	3.17 ± 0.81	53.16 ± 3.56
*F* value		3.601	3.475	2.927
*P* value		0.032	0.036	0.001

The article "Serum Expression of ESM-1, HMWA, and AGEs and Its Relationship with Disease Severity in Patients with Gestational Hypertension" was retracted in 2023. Reasons: signs of a paper mill; compromised peer review; unreliable results or conclusions.

**Table 3:** Correlation analysis of serum ESM-1, HMWA, and AGEs and the degree of gestational hypertension.

Project	Disease severity	
	*r* value	*P* value
ESM-1	0.259	0.002
HMWA	-0.341	0.001
AGEs	0.419	0.001

**Table 4:** Value analysis of serum ESM-1, HMWA, and AGEs to predict hypertension during pregnancy.

Project	AUC (95% CI)	The logo is wrong	*P*	Sensitivity	Specificity	Cut-off value
ESM-1	0.701 (0.603~0.799)	0.050	0.001	81.52	86.59	1.14 *μ*g/l
HMWA	0.652 (0.565~0.739)	0.045	0.001	84.15	87.58	4.33 ng/ml
AGEs	0.982 (0.967~0.998)	0.008	0.001	85.35	88.28	44.87 ng/ml
Joint detection	0.992 (0.983~1.000)	0.005	0.001	89.67	91.24	—

## Data Availability

The data used to support this study are available from the corresponding author upon request.
